This article has been retracted.

# Effectiveness of Proanthocyanidin plus Trimetazidine in the Treatment of Non-Small-Cell Lung Cancer with Radiation Heart Injury

**DOI:** 10.1155/2022/2338622

**Published:** 2022-06-03

**Authors:** Hang Yin, Yue Zhao, Yucui Sun, Jia Liu, Yingjun Han, Zhentao Dai

**Affiliations:** ^1^Ward I, Department of Cardiovascular Medicine, Cangzhou People's Hospital, Cangzhou, China; ^2^Department II of Radiotherapy, Cangzhou Central Hospital, Cangzhou, China

## Abstract

This study was intended to explore the effect of proanthocyanidin (PC) combined with trimetazidine in non-small-cell lung cancer (NSCLC) with radiation-induced heart damage (RIHD). It was a prospective randomized controlled study that 86 NSCLC patients with radiation treatment in Cangzhou People's Hospital from January 2019 and June 2021 were enrolled and randomized to either the control group or the study group via the random table method, 43 cases in each group. The control group received trimetazidine, and the study group additionally received PC. The incidence of RIHD-related clinical manifestation, RIHD-related ECG, and RIHD-related cardiac ultrasound change were all lower in the study group. After radiotherapy, the serum level of superoxide dismutase (SOD) was higher, and malondialdehyde (MDA) was lower in the study group when compared with the control group. After radiotherapy, the serum levels of brain natriuretic peptide (BNP), cardiac troponin (cTnT), creatine kinase (CK), and creatine kinase isoenzymes (CKMB) were all lower in the study group when compared with the control group. The efficacy of PC plus trimetazidine for NSCLC with RIHD is superior to trimetazidine alone, and it significantly mitigates radiation-induced inflammatory response and oxidative stress.

## 1. Introduction

As a major technique to control the occurrence and development of non-small-cell lung cancer (NSCLC), radiotherapy is susceptible to multiple factors such as anatomical location [1, 2]. As a result, the heart is a vulnerable organ, and radiation-induced heart damage (RIHD) is prevalent during radiotherapy of NSCLC and a leading cause of nontumor death [3, 4]. Evidence shows that the risk of cardiac events after three-dimensional radiotherapy appears to be raised by 17.4% as the average cardiac dose of patients increases by 1 Gy [5]. Despite the advancement of radiation treatment and operation techniques, the risk of cardiac events cannot yet be completely eliminated [6].

Currently, drugs are confirmed as an effective way to prevent NSCLC combined with RIHD [7]. Trimetazidine is a commonly used clinical drug for the treatment of coronary dysfunction, myocardial infarction, and angina pectoris by regulating myocardial energy metabolism, inhibiting myocardial fibrosis, and repairing myocardial damage [8–10]. PC, a general term for polyphenols widely existing in plants, is an effective ingredient in traditional Chinese medicine [11, 12]. PC has strong antioxidant and free radical elimination effects, which can effectively eliminate superoxide anion free radicals and hydroxyl free radicals and protect lipids from peroxidation damage [13]. In addition, procyanidins can significantly regulate blood lipids and improve lipid disorders, fight oxidation and clear free radicals, promote vasodilation, and inhibit the production of various inflammatory factors and inflammatory reactions, thus protecting the cardiovascular system [14]. Accordingly, the principal objective of the present study was to investigate the efficacy of PC plus trimetazidine in NSCLC combined with RIHD.

## 2. Methods and Materials

### 2.1. Study Design

It was a prospective randomized controlled study that 86 NSCLC patients with radiation treatment in Cangzhou People's Hospital from January 2019 and June 2021 were enrolled and randomized either to the control group or to the study group, 43 cases in each group. This study has obtained the approval of the Cangzhou People's Hospital Ethics Committee (approval no. 79971) prior to commencing the enrollment.

### 2.2. Inclusion and Exclusion Criteria

Inclusion criteria were as follows: (1) patients who were diagnosed by puncture or surgical pathological examination and were in line with the indications for radiotherapy; (2) combined with RIHD; (3) no abnormal liver and kidney function; and (4) patients and their families were informed of this study and signed the consent form.

Exclusion criteria were as follows: (1) those who received targeted therapy or chemotherapy concurrently; (2) those with serious history of heart disease; (3) those who were allergic to PC or trimetazidine drugs; and (4) the expected survival time was less than half a year.

### 2.3. Treatment Method

All patients received conventional radiotherapy according to their condition. The control group received trimetazidine before radiotherapy (20 mg, Ruiyang Pharmaceutical Co., Ltd., SFDA approval no.: H20066534), 3 times/day, 1 tablet/time; the study group additionally received PC capsules (300 mg/capsule, Shenzhen Hanrong Industrial Development Co., Ltd., SFDA approval no.: G20050295) orally on this basis, 1 capsule/day; all drugs were stopped until the end of radiotherapy.

### 2.4. Clinical Outcome

#### 2.4.1. Primary Outcome

The RIHD is diagnosed by clinical manifestation, ECG, and cardiac ultrasound. Clinical manifestations are chest tightness, chest pain, palpitations, fatigue, etc. Patients with the above symptoms during treatment, or aggravated symptoms, are recorded as positive; otherwise, they are considered negative. ECG includes arrhythmia, ischemic ECG changes, and myocardial infarction ECG manifestations. If the patient's electrocardiogram shows above presentations, or worse than before, it is recorded as positive; otherwise, it is negative. Cardiac ultrasound includes pericardial effusion, abnormal cardiac function, atrial ventricular hypertrophy, and cardiac structural changes such as valve stenosis or regurgitation. At the end of treatment and 3 months after the end of treatment, patients with cardiac ultrasound are considered positive in comparison with those before treatment in the above aspects; otherwise, they are considered negative.

#### 2.4.2. Secondary Outcome

The serum levels of MDA, BNP, BNP, cTnT, CK, CK-MB, or other myocardial markers before and after radiotherapy were measured.

### 2.5. Statistical Analysis

SPSS 22.0 software was used for statistical processing, and GraphPad prism 7 software produced in San Diego was used to plot graphics. The counting and measurement were represented by (*n*, %) and ($\bar{x}\pm s$), respectively, and analyzed by chi-square test and *t* test, respectively. *P* < 0.05 was considered statistically different.

## 3. Results

### 3.1. Baseline Data

The gender, age, smoking history, chemotherapy history, and the percentage of hypertension and diabetes between the two groups were comparable with no significant difference (Table 1).

### 3.2. RIHD-Related Clinical Manifestation

In the control group, there were 4 cases of chest tightness, 2 cases of chest pain, 4 cases of palpitations, and 6 cases of fatigue, with the total incidence of 37.21% (16/43). In the study group, there were 2 cases of chest tightness, 1 case of chest pain, 2 cases of palpitations, and 2 cases of fatigue, with the total incidence of 16.28% (7/43), which was lower than the control group (*P*=0.028), as shown in Table 2.

### 3.3. RIHD-Related ECG

In the control group, there were 14 cases of arrhythmia, 4 cases of ischemic change, and 2 cases of myocardial infarction change, with the total incidence of 46.51% (20/43). In the study group, there were 5 cases of arrhythmia, 4 cases of ischemic change, with the total incidence of 20.93% (9/43), which was lower than the control group (*P*=0.012), as shown in Table 3.

### 3.4. RIHD-Related Cardiac Ultrasound Change

In the control group, there were 6 cases of hydropericardium syndrome, 4 cases of reduced EF, 2 cases of myocardial hypertrophy, and 3 cases of valve disorder, with the total incidence of 34.88% (15/43). In the study group, there were 3 cases of hydropericardium syndrome, 1 case of reduced EF, and 1 case of valve disorder, with the total incidence of 11.63% (5/43), which was lower than the control group (*P*=0.011), as shown in Table 4.

### 3.5. Analysis of SOD and MDA

Before radiotherapy, the serum levels of SOD and MDA were comparable between the two groups (all *P* > 0.05). After radiotherapy, the serum level of SOD was higher, and MDA was lower in the study group when compared with the control group (Figure 1).

### 3.6. Analysis of the Marker of Myocardial Injury

Before radiotherapy, the serum levels of BNP, cTNT, CK, and CKMB were comparable between the two groups (all *P* > 0.05). After radiotherapy, the above indicators were all lower in the study group when compared with the control group (Figure 2).

## 4. Discussion

Statistics show that radiotherapy is associated with the higher incidence of heart disease and risk of death [15]. In essence, RIHD is positively correlated with the dose and volume of radiotherapy [16]. The innovation of radiotherapy technology, especially the use of intensity modulated radiation therapy (IMRT) technology, has tremendously reduced the radiation dose and volume of the heart, yet even low-dose radiation causes heart damage [17]. Moreover, the overall improvement effect of IMRT on radiotoxicity is not remarkable. Trimetazidine is an antiischemic myocardial injury drug widely used in clinical practice in recent years. It reduces the oxidation rate of free fatty acids, controls the energy supply balance of free fatty acid/glucose oxidation, and reduces the demand for oxygen during the production of high-energy phosphate, thereby maintaining the production of ATP and the energy metabolism and contraction function of ischemic myocardial cells and protecting the myocardium [18]. Previous studies used the drug to treat myocardial damage and found that trimetazidine can effectively alleviate the progression of atherosclerotic plaque and prevent myocardial dysfunction [19, 20]. Studies pointed out that the structural types and quantities of PC continue to increase, with a wide range of natural sources and strong biological activity, especially in the prevention and treatment of cardiovascular diseases, reduction of blood lipid, blood pressure and blood glucose levels, and anticancer [21]. With good biological activity, PC have potential prospects in the fields of medicine, food, cosmetics, etc., as a substance with wide distribution in nature, food-borne, strong activity, and low toxicity [22]. In order to alleviate the heart damage induced by radiotherapy for patients with NSCLC, our hospital attempted to treat NSCLC and RIHD with PC plus trimetazidine and produced a satisfactory outcome.

The present study showed that patients who received trimetazidine alone displayed poor electrocardiogram and a higher incidence of abnormal cardiac events than the patients who received the combined treatment. The myocardial markers and SOD levels of the patients after treatment were improved as compared with the baseline values, and the indicators of the study group after treatment were superior to those of the control group. Moreover, the MDA of patients in the study group were considerably lower when compared with that in the control group. All these results indicate that trimetazidine has significant antiischemic properties, which can alter energy substrate metabolism by inhibiting terminal enzymes in the *β*-oxidation pathway, enhance glucose metabolism, and reduce myocardial damage and oxidative stress [23, 24]. It is acknowledged that radiation can induce myocardial cell fibrosis, cause myocardial ischemia and hypoxia, and further lead to myocardial cell apoptosis. As previously noted, trimetazidine can reduce the levels of lactate dehydrogenase, CK-MB, reactive oxygen-free radicals, and MDA in plasma to increase SOD and glutathione peroxidase levels, thereby protecting myocardial cells [25]. Promisingly, the current study confirms the robust efficacy of PC plus trimetazidine on NSCLC combined with RIHD.

## 5. Conclusion

The combination of PC and trimetazidine is a reliable approach to treat NSCLC complicated with RIHD by inhibiting radiation-induced inflammatory response and oxidative stress response.

## Figures and Tables

**Figure 1:** Analysis of SOD and MDA. (a) The serum level of SOD before radiotherapy, (b) the serum level of SOD after radiotherapy, (c) the serum level of MDA before radiotherapy, and (d) the serum level of MDA after radiotherapy. ^*∗∗∗*^indicates *P* < 0.001.

**Figure 2:** Analysis of the marker of myocardial injury. (a) The serum level of BNP before radiotherapy, (b) the serum level of BNP after radiotherapy, (c) the serum level of cTNT before radiotherapy, and (d) the serum level of cTNT after radiotherapy. (e) the serum level of CK before radiotherapy, (f) the serum level of CK after radiotherapy, (g) the serum level of CKMB before radiotherapy, and (h) the serum level of CKMB after radiotherapy. ^*∗∗*^indicates *P* < 0.01 and ^*∗∗∗*^indicates *P* < 0.001.

**Table 1:** The general data.

	Control group (*n* = 43)	Study group (*n* = 43)	*χ* ^2^	*P*
Gender (male/female)	25/18	28/15	0.443	0.506
Age (years)	61.33 ± 9.22	59.14 ± 8.64	1.137	0.259
Smoking history (yes/no)	19/24	17/26	0.191	0.662
Chemotherapy history (yes/no)	22/21	25/18	0.422	0.516
Hypertension (yes/no)	24/19	21/22	0.420	0.517
Diabetes (yes/no)	17/26	15/28	0.199	0.655

**Table 2:** RIHD-related clinical manifestation (*n*, %).

	*n*	Chest tightness	Chest pain	Palpitations	Fatigue	Total
Control group	43	4	2	4	6	16 (37.21)
Study group	43	2	1	2	2	7 (16.28)
*χ* ^2^	4.807					
*P*	0.028					

**Table 3:** RIHD-related ECG (*n*, %).

	*n*	Arrhythmia	Ischemia	Myocardial infarction	Total
Control group	43	14	4	2	20 (46.51)
Study group	43	5	4	0	9 (20.93)
*χ* ^2^	6.295				
*P*	0.012				

**Table 4:** RIHD-related cardiac ultrasound (*n*, %).

	*n*	Hydropericardium syndrome	Reduced EF	Myocardial hypertrophy	Valve disorder	Total
Control group	43	6	4	2	3	15 (34.88)
Study group	43	3	1	0	1	5 (11.63)
*χ* ^2^	6.515					
*P*	0.011					

Note: EF = ejection fraction.

## Data Availability

All data generated or analysed during this study are included in this published article.
